# Biophysical Model: A Promising Method in the Study of the Mechanism of Propofol: A Narrative Review

**DOI:** 10.1155/2022/8202869

**Published:** 2022-05-17

**Authors:** Zhen Li, Jia Liu, Huazheng Liang

**Affiliations:** ^1^Department of Anesthesiology and Perioperative Medicine, Shanghai Fourth People's Hospital, School of Medicine, Tongji University, Shanghai 200434, China; ^2^Translational Research Institute of Brain and Brain-Like Intelligence, Shanghai Fourth People's Hospital, School of Medicine, Tongji University, Shanghai 200434, China; ^3^Clinical Research Center for Anesthesiology and Perioperative Medicine, Tongji University, Shanghai 200434, China; ^4^School of Computer Science and Engineering, Nanjing University of Science and Technology, Nanjing 210016, China

## Abstract

The physiological and neuroregulatory mechanism of propofol is largely based on very limited knowledge. It is one of the important puzzling issues in anesthesiology and is of great value in both scientific and clinical fields. It is acknowledged that neural networks which are comprised of a number of neural circuits might be involved in the anesthetic mechanism. However, the mechanism of this hypothesis needs to be further elucidated. With the progress of artificial intelligence, it is more likely to solve this problem through using artificial neural networks to perform temporal waveform data analysis and to construct biophysical computational models. This review focuses on current knowledge regarding the anesthetic mechanism of propofol, an intravenous general anesthetic, by constructing biophysical computational models.

## 1. Introduction

Propofol is a short-acting intravenous anesthetic commonly used for induction and maintenance of general anesthesia, sedation for adult Intensive Care Unit (ICU) patients. It takes about two minutes to achieve the maximum effect after intravenous injection, and the effect lasts for five to ten minutes. Propofol has been used in clinical anesthesia for more than 30 years. It is widely accepted that improper use of propofol could lead to injection pain, respiratory depression, and circulatory inhibition. Injection pain is the most common adverse reaction of propofol, which mainly comes from the stimulation of blood vessel walls during intravenous injection of the drug. However, the pain will disappear when the patient is sedated, and the pain at the injection site will not be felt when the patient wakes up. Respiratory suppression is one of the severe complications that limit the broader use of propofol. The application of propofol would slow down the respiratory rate and amplitude of patients and sometimes lead to respiratory arrest in severe cases. If the anesthesiologists could not reasonably control the dosage and indication of propofol and continuously monitor the patient's vital signs, the patient's life will be in danger at any time. Another fatal side effect of propofol is circulatory inhibition. Propofol not only has a sedative effect, but also has an inhibitory effect on the circulatory system. Excessive use of propofol could lead to blood pressure drop, arrhythmia, and so on. If there is no continuous electrocardiogram (ECG) monitoring, the patient's life will be at risk. Therefore, the monitoring system of propofol delivery based on the mechanism of this drug is particularly urgent for safe and proper usage. However, the mechanism of propofol remains ambiguous. A large number of research articles have reported that propofol produces general anesthesia through regulating a variety of neural transmitters [1] and ion-channels [2–4]. However, the detailed mechanism underlying the anesthesia effect of propofol on interactions among different neurons in each layer of brain regions remains largely unknown. Therefore, it is demanding to clarify the detailed anesthetic mechanism of propofol. Previous studies have investigated the mechanism of general anesthesia from six aspects, which are molecular [5], synaptic [6], cellular, neural microcircuit [7], systematic (brain regions), and behavior levels [8]. It is well known that these neural networks are comprised of a number of neural circuits that are involved in the anesthetic mechanism [9]. This review focuses on current knowledge in the anesthetic mechanism of propofol using biophysical modeling.

## 2. Propofol May Produce General Anesthesia by Inhibiting Thalamic Rhythm

General anesthesia is a process in which patients go through awareness, sedation, and arousal upon receiving anesthetics. The mechanism of general anesthetics has been one of the most important topics for scientists since its appearance in 1846. The last few decades have witnessed a surge in the discovery of the mechanism of general anesthetics [10–14]. The theory of network regulation in the mechanism of general anesthesia based on neural microcircuit and systematic levels (brain regions) has been the most attractive one among all hypotheses [15]. Alkire et al. used slow imaging methods such as Positron Emission Computed Tomography (PET) and statistical parametric mapping (SPM) to study anesthesia-induced loss of consciousness and to describe dramatic changes in the brain activities. They found that the thalamus became relatively inactive during general anesthesia and named the “thalamic consciousness switch” [16–19]. Ching et al. found that the thalamus was not completely inactive during general anesthesia, which is contrary to the classical theory. Instead, some subsets of the thalamus consolidated their activities into a highly structured *α*-rhythm [20]. These confirmed that propofol may take the anesthetic effect by inhibiting the thalamic rhythm [21, 22].

Propofol also inhibits auditory signal transduction through inhibiting the thalamic rhythm. Purdon et al. found that propofol induced characteristic changes in neural physiological activities in patients and simultaneously inhibited auditory signal transduction [23]. Using functional Magnetic Resonance Imaging (fMRI) and electroencephalogram (EEG), they found that as the dosage of propofol increased, the correct response observed in the auditory tone discrimination task gradually decreased, followed by a complete disappearance of the correct responses and a decrease in activities of the secondary auditory cortex, with activities of the primary auditory cortex unchanged. This demonstrated that general anesthetics could induce loss of consciousness as well as inhibition of auditory transduction in the subjects [24]. The underlying mechanism of propofol inhibiting auditory signal transduction may lie in that propofol enhances GABA_A_ receptor function or GABAergic neurotransmission possibly by facilitating the binding of GABA_A_ receptor to GABA [25, 26]. Inhibitory synapses such as GABA_A_ ligand-gated channel are necessary and sufficient for the synchronization of gamma rhythm [27]. This is consistent with the results of Paik and Wang in that neural networks comprised of inhibitory interneurons are the key element in generating this high-frequency rhythmic activity of gamma oscillation [28, 29]. Experiments on animals and humans using EEG, intracranial EEG (iEEG), magnetoencephalography (MEG), and other techniques have demonstrated that synchronized gamma oscillation is related to auditory sensation [30]. Gamma oscillation is present in a variety of brain regions of mammals and humans, such as the thalamus, somatosensory cortex, and the hippocampus [31]. Although we have learned much about the molecular mechanism of propofol, little is known about the neural mechanism of inhibiting auditory signal transduction [32]. This could be solved through combining studies of neural circuits and biophysical computational modeling. Lee et al. demonstrated neural circuits between cortex layers and cortical areas could be coordinated and schemed by brain rhythms [33], which adds evidence to the theory of propofol inhibiting auditory transduction by modulating gamma oscillation.

## 3. The Role of Computational Modeling in the Study of the Neural Mechanism of Propofol

As a result of the rapid development in modern informatics tools, research on brain structure and function has been surging by combining neuroscience and bioinformatics tools [34–39]. For example, it is possible to complete the mesoscopic mapping of neural circuits and their activity patterns and to explore the underlying mechanism in animal models [40–46]. This also applies to research on the mechanism of propofol with the assistance of computational modeling [47]. Ching et al. found that the *α*-rhythm induced by propofol was related to loss of consciousness. They built a thalamocortical model to simulate the effect of propofol by combining it with the known cortical dynamics and thalamus models [48]. They also found that the state of consciousness of patients was closely related to the highly structured EEG produced by propofol and the highly structured brain rhythmic activities can be simulated using dynamic system models [20]. They discovered that propofol might act on GABAergic neural networks in the cortex, thalamus, and the brainstem to induce profound brain dynamics which then led to changes from sedation to loss of consciousness. Due to the participation of the thalamus, synchronous rhythms produced by the cerebral cortex may prevent responses to external stimuli, thus maintaining an unconscious state.

Lee et al. simulated interactions between the primary auditory cortex (A1) and the secondary somatosensory cortex (Par2) as observed in vitro by constructing a biophysically based computational model [33]. They proposed that one of the most important factors influencing the gating process that regulates the bottom-up sensory signaling from A1 to Par2 is the coordination between the top-down gamma [14] and beta rhythms. This coordination was regulated by cholinergic modulation between the cortices. This sets a good example of studying the mechanism of propofol using biophysical computational modeling.

## 4. Biophysical Modeling and Computational Simulation Are Important Methods in Studying Neural Networks

It is difficult to investigate the mechanism of interactions within and between neural networks, due to the complexity of the biological neural networks and the limitations of experimental conditions. The rapid development of information technology endowed researchers to examine biological neural networks using diverse techniques, not relying on biological experiments alone [49–52]. To study neural networks under various conditions, mathematical modeling and computer simulation can be easily used to simulate the dynamic processes of various neurons and brain regions, especially to describe the electrophysiological activities of individual or collectively recorded neurons in large neural networks. Neuroscience deciphers the function of the brain from all aspects of the brain, such as the interaction between molecules and their relationship with behavior. Mathematical methods and statistical ideas play an important role in explaining and analyzing a variety of phenomena of the brain. Advances in measurement and storage devices have also made it possible to record the electrical activity of neurons in detail, which consequently help neuroscientists better deal with large experimental databases.

In the 1950s, Hodgkin and Huxley had studied the ionic current in the squid giant axon [53]. Through a series of well-designed experiments, they found why the current generation is the conductivity change of the calcium and potassium channels in the axon membrane. They established the classical Hodgkin-Huxley model (i.e., H-H model) describing the conductivity of calcium and potassium varying over membrane potential as well as time. This model accurately predicted the temporal evolution of membrane conductance, the shape of the action potential, morphological changes of the action potential with sodium concentrations, the number of sodium ions involved in the inward flux across the membrane, the propagation speed of the action potential, and the voltage curves of sodium and potassium ions [53, 54]. The H-H model has many extensions in the field of computational neuroscience, including models that capture additional biological features, such as extra ion currents [55] and various aspects of the extracellular environment of neurons [56], both of which introduce new fast and slow time scales to the dynamic equation. Although it is necessary to take the complexity of biological conditions into account and apply more complex mathematical logic to modeling when studying a large number of neuronal activities, the H-H model is still the framework of computational neuroscience [57, 58]. It lays the foundation for electrophysiological modeling. More accurate models describing changes in the membrane potential of neurons were established based on it, such as the calcium-dependent channel model [59], the single-ion channel Markov model [60], the multicompartment model [61], and so on. A synaptic model [62] was also built to describe interactions between neurons. By combining these models, a neural network model can be directly constructed. For example, a multicompartment model is used to describe the cell bodies, axons, and dendrites of neurons, and a synaptic model to connect compartment models. After converting the mathematical model into the corresponding computer algorithm, dynamic changes of the neural network can be simulated.

Based on the models mentioned above, it is common to investigate the gamma-band oscillation by constructing a biophysical computational model. Borgers et al. built a computational model mimicking the local circuit comprised of a few inhibitory and excitatory neurons to demonstrate interactions between cholinergic modulation, gamma-band oscillation, and selective attention [63]. To study the mass phenomenon in the whole thalamus cortex, Traub et al. [58] constructed a computational model including large-scale networks consisting of various neurons. Recently, gamma oscillation in the auditory transmission pathway has drawn extensive attention to investigate this phenomenon. Lee et al. [33] has established a computational model on interactions between the primary auditory cortex and the secondary somatosensory cortex to demonstrate the correlativity between gamma oscillation and information transmission between these two regions. This model can precisely simulate the outcomes of biological experiments and accurately predict experimental phenomena.

Apart from directly simulating biological processes under experimental conditions, the computation models can also be used in clinical scenarios. For example, Recurrent Neural Network (RNN) is a type of special neural network with memory function, which can effectively use time information for time series analysis. The RNN model and its modified form—the Long Short-Term Memory (LSTM) model—are often used to monitor the depth of anesthesia. The traditional RNN model has the problem of gradient disappearance or gradient explosion. The LSTM model, an improved version of the RNN model, can simulate nerve cells by simply adding a number of gates to effectively deal with serial data (see Figure 1) and consequently solve this problem to some extent [64]. Li et al. [65] proposed a method for monitoring the depth of anesthesia based on LSTM and sparse denoising autoencoder (SDAE) combined with EEG signals. Compared with models using a single feature, this model can accurately estimate the depth of anesthesia with a higher probability. Sun et al. [66] developed an RNN model using a clinical dataset of 154 patients undergoing anesthesia. Without any feature extraction, end-to-end training is used to distinguish depth of anesthesia from nonsedation using the original EEG spectrum. Compared with the simple and smooth feedforward model, their RNN model can continuously provide a better and reliable estimation of the sedation level.

## 5. Artificial Intelligence (AI) and Anesthesia Optimization

The application of artificial intelligence in medical and health field is expanding rapidly, including image recognition, new drug research and development, medical robot, assistant diagnosis, and so on. As a data-intensive discipline, anesthesiology has natural advantages in the application of AI, including the evaluation of anesthetic depth, the construction of predictive models, the establishment of clinical decision support tools, and intelligent drug delivery system. The health data of patients before and after operation and a large number of monitoring data produced during operation are the basis to guide anesthesiologists to judge the state of anesthesia and prevent adverse events, but it is often difficult for the differences in individual patients and medical conditions to achieve accurate management of each patient, which is the main cause of anesthesia and perioperative complications and even death. One of the advantages of AI is that it has strong data processing ability and self-learning ability. Through machine learning, we can effectively integrate and deal with the complicated clinical big data and summarize the rules, so as to optimize the anesthesia strategy to achieve accurate anesthesia. The accurate monitoring of anesthesia depth/state can be achieved by integrating perioperative monitoring data based on AI convolutional neural network modeling. Sadrawi [67] et al. take the subjects' EEG, EMG, heart rate, blood pressure, pulse, and signal quality index as input signals through machine learning. The artificial neural network model can monitor the depth of anesthesia significantly higher than the existing depth of anesthesia monitoring. Saadeh [68] et al. have further improved the anesthetic depth monitoring system based on AI analysis EEG, which can be used under harsh conditions such as different ages and different drugs, with an accuracy of 92.2% and a delay time of only 1 s, which can more accurately reflect the depth of anesthesia. Secondly, the clinical decision support system and anesthetic closed-loop system constructed on this basis can help to achieve accurate anesthesia and optimize anesthesia management, thus greatly reduce the workload of anesthesiologists. Ultrasound-guided nerve block is an important technical means of precision anesthesia, but because of its complexity and diversity, it is difficult to guarantee the popularity and blocking effect. Bowness et al. [69] built a clinical support system for nerve block based on AnatomyGuide system by learning from big data, which can effectively assist clinicians to identify nerve block and operate and achieve the role of optimizing anesthesia management. During general anesthesia, a number of studies have shown that closed-loop management based on anesthetic depth can more safely guide clinical anesthetic drugs to achieve accurate anesthesia. During the perioperative period, anesthesiologists need to collect and measure the management of blood glucose, blood pressure, and cardiac output. The complicated process of judgement and regulation is often lagging, while the subjournal Lancet [70] reports that perioperative closed-loop insulin based on deep learning and norepinephrine management system can optimize the existing anesthetic regimen from multiple dimensions and eliminate the possibility of human error. It could also provide a better clinical approach to improve the prognosis of patients. In addition, one of the challenges faced by anesthesiology is that the prediction and management of perioperative adverse events, such as hypoxemia, hypotension, etc., will cause a certain degree of damage to the brain and peripheral organ function of patients and even death. The machine learning model developed by Lundberg et al. [71] could predict the impending hypoxemia more accurately than anesthesiologists and point out the causes of hypoxemia, with early prediction of perioperative adverse reactions and early notification of intervention by anesthesiologist. This can not only improve the efficiency of preoperative evaluation of anesthesiologists, but also optimize the perioperative patient management and ensure the perioperative safety of patients. AI has also been continuously developed in the field of anesthesia and perioperative medical transformation. McGill University in Canada has developed the first Kepler remote artificial intelligence intubation system through the combination of video laryngoscope and robotic arm. With the help of AI, anesthesiologists can not only fully understand the past clinical diagnosis and treatment information of patients and carry out rapid preoperative evaluation, but also use AI to dig out more hidden information and improve postoperative outcome. Cheng et al. [72] automatically assessed infant pain through machine learning of facial expressions. Lee et al. [73] found that changes in autonomic nerve activity in the human body are highly related to the degree of pain through functional Magnetic Resonance Imaging (fMRI) and AI technology. Doctors can score pain for patients who are unable to communicate by monitoring autonomic nerve activity, with an accuracy of 92.4%, greatly reducing the possibility that such patients will be converted into chronic pain after operation.

## 6. Evidence in Biological Neural Networks Promotes the Development of Computational Science

With the advance of computer science, the biological processes can be simulated and the behaviors of neurons efficiently explored in the computer. Similarly, simulating the biological process can promote the development of computer science, especially in the field of information processing and artificial intelligence. Artificial neural network [74–77] is a type of information processing and analysis algorithm inspired by the biological neural system. It imports the information processing of neurons into simple models based on data analysis and forms a network structure by using a weighted synaptic connection [78–83]. This model plays an important role in the application of information processing, including machine learning [84–86], computer vision [87–89], biological and medical data analysis [90, 91], and so on. In biomedicine, artificial neural networks are especially important as they can overcome difficulties in the detection and analysis of biological signals [92], signal processing, and recognition of medical images [93], which remain a challenge for conventional methods [94]. Compared with real-life neural modeling, artificial neural network modeling is much simpler and more direct. Take the widely used multilayer perceptron as an example; the basic module in multilayer perceptron is artificial neurons [95] which is composed of weighted synapses and nonlinear activation. In real neurons, the activation of them depends not only on the weighted sum of signals. But the simple weighted sum can fit any functions in theory when they are connected layer by layer.

In addition, there are some models based on the lateral inhibition of the primary visual cortex, such as self-organizing mapping [96, 97], cyclic neural networks [98], the Hopfield network [99, 100], and so on. With the in-depth study of the information processing mechanism of the human brain, it has been found that sensory information is expressed through complex hierarchical structures, such as the V1∼V5 areas of the visual cortex. Visual information is transmitted and processed layer by layer before being consolidated into advanced perception and memory. Inspired by this type of information processing, deep neural networks were developed by constructing hierarchical information processing layers [101, 102]. This network model has better information processing and modeling ability than the shallow network model and can directly learn the input data without the process of data preprocessing and feature extraction [103, 104]. Thus, it can be applied to various scenarios such as speech recognition [105], natural language processing [106], image/video processing [107], and so on. Currently, there are a decent number of models in the field of deep neural networks, for example, the convolutional neural network [108, 109] inspired by the receptive field in the visual cortex, the sparse representation models [110, 111] simulating the V1 and V2 in the visual cortex, and so on. However, due to the lack of knowledge and understanding of the mechanism of biological neural networks, these models are simply mimicking the characteristics of local neurons that are observed with current techniques. They only simulate part of the evidence in real neural systems. For example, convolutional neural network uses the convolutional kernels to imitate the receptive field while ignoring many biological details. For convenient optimization in practice, many sparse representation models simulate the sparse regions by using differentiable functions. With the increase of data volume and complexity, it is one of the challenges for the field of artificial intelligence to build a more efficient information processing model through learning from the biological nervous system.

Though brain-inspired learning models are successful in simulating the learning mechanism of the biological neural system and processing practical information, they are simply designed based on mathematic theories to efficiently work on computational devices. With the development of hardware, especially of the Graphics Processing Unit (GPU) and corresponding parallel computation methods [112, 113], more complex models that are closer to the real neural system have been developed. The most popular learning model deep neural networks [101, 114] are inspired by the hierarchical architecture of brain learning. In contrast to simulating models, such as the abovementioned H-H model, they aim to simulate the real neural system as true as possible to explore the behaviors of the neural system. The common problem these two types of models encounter in practice is the low computational efficiency. Due to the limitation of computational capacity, the simulated model only contains a small number of neurons. Undoubtedly, simulating a more complex system will result in more interesting findings. Inspired by the development of information models, more complex models can construct a high-performance computational device. It might be a new direction for simulating modeling to study the mechanism of propofol with the assistance of new computational platforms such as GPU parallel computation.

## 7. Conclusions and Perspectives

In the study of propofol, most computational simulation models focus on a small local network with several neurons. For more neurons and more complicated neural networks, traditional models may fail to efficiently simulate them. To overcome this difficulty, brain-inspired information processing models may provide solutions. On one hand, parallel computation based on GPU has significantly increased the capacity of artificial intelligence models. Similarly, the simulating models can also be executed based on parallel computational platforms. Since the structure of neurons is distributed, each neuron can be simulated in an arithmetic unit and updated parallelly by using parallel computation. In theory, the computational complexity of parallel computation increases linearly with the increase of neurons. For serial computation, the computational complexity even increases exponentially. As a result, much more complex structures and more types of neurons can be efficiently simulated. On the other hand, artificial intelligence models provide excellent modeling methods for simulating real neurons. The widely used H-H model successfully simulates the input and output relationship of a neuron as shown in Figure 2. The parameters are estimated based on data collected from in vivo experiments. However, there are numerous types of neurons in the brain; it is difficult for a model to simulate all of them. The input and output relationship can also be learned by artificial intelligent models, such as the abovementioned artificial neural networks. In theory, a two-layer neural network can model any function. As shown in Figure 3, the RNN model is adept in dealing with time series data which can be used to simulate the function of neurons. The parameters within the RNN are learned from data collected from in vivo experiments. Each neuron can be simulated through learned RNNs. Furthermore, with the multidimensional modeling capacity of neurons, one neural network can also simulate a group of neurons, such as a local cortical area. Therefore, a larger region in the brain can be simulated with numerous artificial neural networks.

Propofol produces general anesthesia by inhibiting the thalamic rhythm, which is achieved through the participation of neural networks comprised of multiple neural circuits. Among the many methods to study the anesthetic mechanism of propofol, computational modeling can help to find changes in the brain rhythm upon injection of propofol, which facilitates our understanding of the anesthetic mechanism of propofol. This will guide the safe and rational use of propofol clinically.

## Figures and Tables

**Figure 1:** Model structure of biological experimental data analysis. “Cell” represents the cell body and consists of three gates. The input gate (Input Gate), the output gate (Output Gate), and the amnesia gate (forget gate) are used to control the memory and forgetting of time series data. The S-shaped curve represents the activation function, and the black dot represents the data operation. The model can use “forget gate” to choose the state information before forgetting, to maintain useful information to complete the analysis of time series.

**Figure 2:** Construction process of the H-H model. In essence, the construction of a simulating model is the process of curve fitting by assuming the model and estimating parameters within it. The H-H model assumes an equivalent circuit which is represented by the differential equation. There are a number of parameters in the model that have to be estimated to fit the membrane potential as recorded in experiments in vivo. For different types of neurons, the parameter sets are also different but they follow the same modeling process.

**Figure 3:** Learning process of the RNN for simulating. Some artificial neural network models can also be used to model neural activity after training by the data generated from in vivo experiments. This figure shows an example of the modeling process for the RNN. To explore the effect of propofol on the auditory cortex, in vivo experiments are completed and the neural network model such as the RNN is trained using experimental data. Then the network is used to simulate the input and output relationship of different types of neurons. By constructing the neurons in a network, the system can be effectively simulated.

## Data Availability

The data that support the findings of the study are available from the corresponding author upon reasonable request.
